The article "Comparative Analysis of the Efficacy of Transurethral Bipolar Plasma Needle Electrode and Ring Electrode in the Treatment of Non-Muscle-Invasive Bladder Cancer" was retracted in 2023. Reasons: signs of a paper mill; compromised peer review; unreliable results or conclusions.

# Comparative Analysis of the Efficacy of Transurethral Bipolar Plasma Needle Electrode and Ring Electrode in the Treatment of Non-Muscle-Invasive Bladder Cancer

**DOI:** 10.1155/2022/6044676

**Published:** 2022-05-13

**Authors:** Pei Zheng, Jianhua Zhang, Yahong Zhu, Xiaodong Guan, Jianwen Quan, Qi Li, Fen Yi

**Affiliations:** Yuncheng Central Hospital, Yanhu District, Yuncheng, Shanxi Province, China

## Abstract

Bladder cancer is the most prevalent tumor of the urinary tract, ranking seventh in males and seventeenth in women. The gold standard for the definitive diagnosis and initial treatment of non-muscle-invasive bladder cancer is transurethral resection (TUR) of the bladder tumor. The ability to accurately detect disease, typically in the presence of hematuria as well as to detect early recurrent tumors in patients with a history of NMIBC, is critical to the successful treatment of non-muscle-invasive bladder cancer (NMIBC). Unfortunately, the current biomarker landscape for NMIBC is still evolving. Cystoscopy remains the gold standard, but it can still miss 10% of tumors. As a result, physicians frequently employ additional diagnostic tools to aid in the diagnosis of bladder cancer. The efficacy of transurethral bipolar plasma needle electrodes and ring electrodes in the treatment of non-muscle-invasive bladder cancer was compared and analyzed in this study. During our study, 100 patients with non-muscle-invasive bladder cancer admitted to our hospital between June 2019 and June 2020 were randomly assigned to a control group and an observation group, with 50 cases in each group. The observation group was given a bipolar plasma needle electrode, while the control group was given a bipolar plasma ring. Patients continued to receive bladder irrigation chemotherapy as well as traditional Chinese medicine (TCM) treatment as part of our treatment plan, while the control group received only bladder irrigation chemotherapy. Clinical factors such as operational blood loss, catheter indention time, length of hospital stay, and others were compared between the two groups. When the risk grades in the two groups were compared, the observation group had fewer medium- and high-risk grades than the control group, but the control group had more low-risk grades, with statistical significance (*P* < 0.05).

## 1. Introduction

Bladder cancer is the 30^th^ most deadly and 10^th^ most common type of cancer in the world. The affection rate of this deadly disease is more in men as compared to women. In China, bladder cancer still has the greatest rate of tumors in the urinary reproductive system. Its incidence is rising steadily, especially in Europe and other developed countries [1]. Approximately, 75% of BCs do not involve the muscle wall of the bladder and are called non-muscle-invasive bladder cancer (NMIBC) [2]. Urothelial cell carcinoma is the most frequent pathological kind of bladder cancer, which can be classified as non-muscle-invasive or muscular-invasive depending on whether it infiltrates into the mucosa [3]. The main treatment for non-muscle-invasive bladder cancer is surgical resection, but the postoperative recurrence rate can be as high as 70%, and about 10% of patients will develop muscular-invasive bladder cancer [4]. The new standard for diagnosing and treating bladder cancers is transurethral resection (TUR). Maximal TUR of bladder tumors (TURBT), defined as macroscopically full resection of the bladder tumor when it is safe to do so, is important to successful therapy in mono- and multimodality regimens [5].

The capacity for disease detection effectively, generally in the presence of hematuria, as well as the early detection of recurring tumors in patients with a history of NMIBC, is critical to the successful treatment of non-muscle-invasive bladder cancer (NMIBC). Cystoscopy, which has survived the test of time and currently, is the gold standard for bladder cancer detection. The sensitivity of cystoscopy is 85–90%, yet it can miss 10% of papillary tumors. The main issue in clinical practice right now is a lack of understanding of the risk of NMIBC. This is generally regarded as a low-grade malignancy with a low rate of carcinoma in situ (CIS), irregular treatment of special histological types of NMIBC, inadequate treatment of high-risk NMIBC, irregular bladder perfusion treatment, and other issues worthy of consideration.

The traditional open cystectomy has been replaced by transurethral minimally invasive technology, of which transurethral tumor resection is the standard surgical method for the treatment of non-muscle-invasive bladder cancer at the moment, with remarkable clinical efficacy [6]. For non-muscle-invasive bladder cancer (NMIBC), transurethral resection of the tumor (TURBT) is the best option [7]. The surgery has two goals: one is to remove all visible tumor tissue, and the other is to grade and stage the malignant degree of the removed tumor tissue [8]. Traditional TURBT, on the other hand, uses annular electrodes to perform layered resection of the tumor, and the excised tissue is relatively small, with each tissue undergoing electrocoagulation and burning, which is not conducive to pathological staging. The greater the contact surface with the tumor, the greater the extrusion pressure, the more bleeding, and the greater the risk of obturator nerve reflex due to bladder perforation [9, 10].

Although these markers are currently available, their modest performance, limited added diagnostic value, increased cost, and lack of an accurately defined role in the course of bladder cancer diagnosis and treatment timeline have limited their widespread use [11]. As a result, there is still a need for more biomarker development and validation in this disease space [12, 13]. The purpose of this study was to investigate the efficacy of transurethral bipolar plasma needle electrode and ring electrode in the treatment of non-muscle-invasive bladder cancer and to provide a foundation for clinical treatment selection.

1. We aimed to compare and analyze the efficacy of transurethral bipolar plasma needle electrode and ring electrode in the treatment of non-muscle-invasive bladder cancer.
2. We compare the changes in magnetic resonance imaging (MRI) images, blood routine, immune function, leukocyte level, and other related indexes before and after treatment between the observation group and control group.
3. We experimentally proved that compared with transurethral bipolar plasma ring electrode, the needle electrode is more effective in the treatment of non-muscle-invasive bladder cancer.

The rest of our paper is given as follows: Section 2 illustrates materials that we have used during our research work.  Section 3 explains our proposed methodology.  Section 4 elaborates on the experimental work.  Section 5 is based on discussion and finally, we conclude our work in Section 6.

## 2. Materials

### 2.1. Objects in Our Research

The Department of Urology, Yuncheng Central Hospital, China, undertook this prospective case-control study from June 2019 to June 2020. We chose 100 patients with non-muscle-invasive bladder cancer who were admitted to our hospital between June 2019 and June 2020. Among them, the total number of female patients was 50 and male patients were also 50. There were 4 cases of complications in the observation group (8.00%), and 15 cases of complications in the control group (30.00%). The incidence of postoperative complications in the observation group was significantly lower than that in the control group, with statistical significance (*P* < 0.05). After therapy, some individuals experienced recurrence, with the number of recurrences ranging from three to more than 35. The Yuncheng Central Hospital Ethics Committee approved and oversaw the study. Patients were enrolled if they matched the inclusion criteria and exclusion criteria.

### 2.2. Inclusion Criteria

The inclusion criteria were as follows:

1. By ultrasonography and cystoscopy, the patient was diagnosed as non-muscle-invasive epithelial carcinoma of the bladder;
2. Age between 18 and 80 years, newly treated patients;
3. Tumor stage ≤ *T*2, no tumor metastasis occurred after examination, and transurethral bipolar plasma needle electrode and ring electrode were used to treat non-muscle-invasive bladder cancer by the whole resection;
4. The bladder cancer did not involve the bladder muscle layer, and there was no lymph node metastasis or distant metastases, according to the imaging results;
5. Subjects who agreed to have a transurethral needle electrode resection or a transurethral holmium laser resection and who can be followed up with routine perfusion treatment after the procedure;
6. Capacity of bladder ≥250 mL;
7. The medical history was complete;
8. Written informed consent given by patients.

### 2.3. Exclusion Criteria

Exclusion criteria were as follows:

1. The tumor diameter was >3 cm;
2. Severe insufficiency of heart, liver and kidney;
3. Urinary tract infection;
4. Complicated with other malignant tumors;
5. With mental illness or communication difficulties;
6. Pregnancy or lactation;
7. Contraindications include pregnant women, critically ill patients, and others with major cardiovascular illness, considerable abnormal coagulation function, non-transitional epithelial tumors that prevent patients from lying flat, urethral stricture, and others;
8. Those who the researchers believe will compromise surgical efficacy and safety evaluations as well as those who have poor compliance;
9. Other unsuitable candidates.

### 2.4. General Information

According to the random number table method, they were divided into the control group and observation group, with 50 cases in each group. There was no significant difference in general data between the two groups (P＞0.05), and the two groups were comparable. All cases signed the informed consent and were approved by the ethics committee of our hospital. The general information about the control group and observation group can be seen in Table 1.

The purpose of this study was to look into the effectiveness of transurethral needle electrode resection and transurethral holmium laser resection for non-muscular-invasive bladder cancer. Patients were enrolled in this study prospectively and were divided into two groups based on the type of surgery.

## 3. Methodology

During our surgical method, we have taken the lithotomic position under epidural or general anesthesia by using an Olympus plasma electroscope. The outer sheath F26.5, 12° observation lens, continuous cleaning with normal saline, Olympus plasma needle electrode WA22355 A, electrocuting power of 280 W, and electrocoagulation of 100 W were used in bipolar mode. The observation group was treated with a bipolar plasma needle electrode, which was applied to ring electro coagulation 0.5 cm away from the tumor for one week. The surgical resection area was marked, and the needle electrode was inserted into the submucosa of the bladder. Short-time excitation, point-like incision, cut-and-coagulant combination, along the superficial muscular layer, using “pick,” “push,” “hook,” and other techniques, gradually complete resection of the tumor. The needle electrode and rolling electrode were used for local exact hemostasis, and the pathological specimens were taken out. For large tumors, they could be separated before being completely separated from the muscle tissue so as to be removed [11].

The control group was treated with a bipolar plasma ring electrode. Similarly, the pathological specimens were removed after the tumor body, and the surrounding basal mass of 2 cm was excised from the tumor surface to the depth of normal muscle tissue. The bladder was examined once more, and there was no evidence of a remnant tumor or ongoing bleeding. The bladder was washed until the urine was clear with an F20 three-chamber urethral catheter [12].

The catheter was routinely wailed after tumor tissue was removed in both groups. The bladder perfusion chemotherapy (1.0 g gemcitabine + 20 ml normal saline) was administered immediately following surgery, with a 30-minute perfusion time. Following that, the bladder was flushed continuously until the urine was clear, and antibiotics were administered to prevent infection after surgery. Later on, bladder perfusion chemotherapy was maintained, once a week for the first eight weeks, then once a month. The total number of bladder perfusion chemotherapy sessions was 18 after 10 consecutive days. Both groups returned to the hospital every three months after the operation for a reexamination to determine the status of recurrence.

### 3.1. Observational Index

Regular measurement and documentation of clinical observations are required for patient assessment and clinical deterioration recognition. The term “objective observation” refers to visible and measurable signs that are usually true. Monitoring and recording vital signs such as breathing, blood pressure, pulse and temperature, input/output ratio, and so on are all part of this. We can compare these readings to previous readings and monitor any changes or progression in the residents' conditions if we keep a consistent and accurate record of them. The following clinical indicators were observed in both groups:

#### 3.1.1. Clinical Indicators

Clinical indicators represent the level of treatment provided to patients. They must meet high-quality criteria and be deliberately and transparently produced. Furthermore, they must be relevant to crucial areas of care quality. There should also be sufficient research proof that the suggestions they are based on are related to clinical effectiveness, safety, and efficiency. Our clinical indicators are excellent for comparing professionals, practices, and institutions since they measure quality legitimately and reliably with minimum inter- and intraobserver variability. Operative blood loss, catheter indention duration, length of hospital stay, obturator nerve reflex rate, depth of pathological specimen, and postoperative recurrence rate during follow-up are the clinical markers in our treatment of non-muscle-invasive bladder cancer.

#### 3.1.2. Risk Grade

Risk grades are a standardized technique to evaluate the volatility of an asset across a variety of asset types. According to the Chinese Guidelines for Diagnosis and Treatment of Urological Diseases (2014) [13], the postoperative tumor risk of two groups was assessed. There were three levels of risk: low risk, medium risk, and high risk.

#### 3.1.3. Immune Function Indicators

Based on several established features, bladder cancer is an ideal disease state for studying immune evasion and mechanisms for improving immune response. These characteristics include distinct molecular/genomic subtypes of bladder cancer, known response rates to currently available immune therapy, and a once-in-a-lifetime opportunity to study treatment response. The percentages of CD4 + T lymphocytes and CD8 + T lymphocytes in the two groups' venous blood before and 2 hours after surgery were calculated, and the CD4 + /CD8+ ratio was calculated. BD FACS CANTO flow cytometry was used to detect CD4 + and CD8 + cells.

### 3.2. Complication Indicators

The rates of postoperative complications such as bladder perforation, obturator nerve reflex, and bladder irritation were compared statistically between the two groups.

### 3.3. Statistical Method

For our work, we have used SPSS 22.0 for statistical analysis. Measurement data were expressed as *x* ± *s*, and counting data were expressed as (%). All tests were two-sided. *P* < 0.05 was considered statistically significant. The results of the two groups were compared using a two-sided *t*-test for continuous variables and a chi-square test for categorical variables. Kaplan–Meier method was used to evaluate the survival data.

## 4. Results

### 4.1. Bladder Cancer Reappearance after Survey

Three cases of recurrence occurred within four months, in both the control and observation groups, and there was no recurrence in the control group. Within 7 months, the control group's recurrence rate was 15.13 percent, whereas the observation group's recurrence rate was 5.2 percent, which was significantly lower than the control group's recurrence rate. Within 10 months, seven cases recurred: three in the observation group (9.2% recurrence rate) and five in the control group (22.5% recurrence rate). This showed that combining Chinese and Western therapy to treat bladder cancer after surgery was beneficial in preventing recurrence.

### 4.2. Results of Clinical Indicators

Clinical parameters were evaluated between the two groups based on the outcomes of our research. Surgical blood loss, catheter indention duration, length of hospital stay, obturator nerve reflex rate, pathological specimen depth, and postoperative recurrence rate during follow-up are some of these. Similarly, the observation group's clinical indicators were lower than the control group's (P0.05).  Table 2 shows the results of clinical indicators:

### 4.3. Results of Risk Grade

The comparison of risk grades between the two groups revealed that the number of medium- and high-risk grades in the observation group was lower than that in the control group with statistical significance (P 0.05). Similarly, the number of low-risk grades was higher in the experimental group than in the control group.  Table 3 displays the risk grade results:

### 4.4. Results of Immune Function Indicators

Before the operation, there was no significant difference in CD4+, CD8+, or CD4+/CD8+ between the two groups (*P* > 0.05). After 2 hours of operation, CD4+, CD4+/CD8+ decreased, and CD8+ increased in the two groups, with a significant (P0.05) difference and the degree of decrease or increase in the observation group was less than that in the control group, with a significant (P0.05) difference.  Table 4 displays the results of immune function indicators:

### 4.5. Results of Complication Indicators

There were 4 complications in the observation group (8.00%) and 15 complications in the control group (30.00%). The incidence of postoperative complications with statistical significance (*P* < 0.05) was significantly lower in the observation group than in the control group.  Table 5 displays the results of the complication indicators:

The contrast between the control and observation groups is depicted in Figure 1. Here, *p* > 0.05 indicates statistical significance, and x2/*t* equals 0.154. The number of cases in the control group is 50, and the number of patients (male = 28 and female = 22) is also 50. Similarly, there are 50 cases in the observation group, with 50 patients (male = 26 and female = 24).

Figure 2 represents the comparison between the control group and observation group based on TNM staging of the tumor (T1 cases and T2 cases), Tumor number (single cases and multiple cases), and American Society of Anesthesiologists (level 1 and level 2). For T1, the control and observation groups are 16 and 18, for T2 they are 34 and 32, for single instances, they are 18 and 17, for multiple cases, they are 32 and 33, and for level 1 they are 26 and 23, and level 2 they are 24 and 27.

The comparison between the control group and the observation group based on risks such as low risk, medium risk, and high risk is shown in Figure 3. It is clear from the figure that the number of medium-risk and high-risk grades in the observation group was lower than that in the control group, while the number of low-risk grades was greater than that in the control group, with statistical significance (*P* < 0.05).

## 5. Discussion

Bladder tumor is the most common malignant tumor in urinary tract tumors, with higher morbidity and mortality, and the incidence in males is higher than that in females [14]. Non-muscle-invasive bladder cancer accounts for about 70% of the primary bladder tumors, including TA, T1, and TIS stages of bladder cancer, which can further progress to muscular-invasive bladder cancer [15]. Radical cystectomy is the main method of choice for the treatment of non-muscle-invasive bladder cancer in clinical practice. It has a good local control effect on the primary tumor, but it also has some problems such as complicated operation, large intraoperative blood loss, long operation time, and high incidence of postoperative complications [16, 17]. Transurethral resection of bladder tumor has long been the “gold standard” for the treatment of non-muscle-invasive bladder cancer [18]. However, with the progress of medical equipment and the continuous practice and understanding of traditional transurethral electric resection of bladder tumors, its limitations have gradually emerged. The limitations of traditional Turbo surgery have been summarized, such as segmented resection, easy obturator nerve reflex, high postoperative recurrence rate, and difficult tumor staging [19]. In recent years, transurethral resection has become more and more accepted [20].

This study showed that clinical indicators were compared between the two groups, including operative blood loss, catheter indention time, length of hospital stay, obturator nerve reflex rate, depth of pathological specimen and postoperative recurrence rate during follow-up, and clinical indicators of the observation group were lower than those of the control group (*P* < 0.05). Comparison of risk grades between the two groups showed that the number of medium-risk and high-risk grades in the observation group was lower than that in the control group, while the number of low-risk grades was greater than that in the control group, with statistical significance (*P* < 0.05). There was no significant difference in CD4+, CD8+ and CD4+/CD8+ between the two groups before operation (*P* > 0.05). 2h after operation, CD4+, CD4+/CD8+ decreased and CD8+ increased in the two groups, the difference was significant (*P* < 0.05), and the degree of decrease or increase in the observation group was less than that in the control group, the difference was significant (*P* < 0.05). There were 4 cases of complications in the observation group (8.00%), and 15 cases of complications in the control group (30.00%). The incidence of postoperative complications in the observation group was significantly lower than that in the control group, with statistical significance (*P* < 0.05).

## 6. Conclusion

Non-muscle-invasive bladder cancer continues to be a major urologic oncologic concern as well as a large financial burden on the healthcare system. In the evaluation of high-risk NMIBC, repeat TURBT is becoming increasingly important. We found that the needle electrode was more successful than the transurethral bipolar plasma ring electrode in the treatment of non-muscle-invasive bladder cancer. The intraoperative blood loss was minimal after needle electrode therapy, the hospital stay could be greatly reduced, the risk level was low, the immune function index value was high, and postoperative problems were minimal. We experimentally demonstrated that when risk grades were compared between the two groups, the number of medium risk and high-risk grades in the observation group was lower than that in the control group, while the number of low-risk grades in the observation group was greater than that in the control group, with statistical significance (P 0.05). Compared with the transurethral bipolar plasma ring electrode, the needle electrode was more effective in the treatment of non-muscle-invasive bladder cancer. After needle electrode treatment, the intraoperative blood loss was small, the hospital stay could be significantly shortened, the risk level was low, the immune function index value was high, and postoperative complications were few. In the future, we hope to apply this approach to other diseases such as heart disease and diabetes.

## Figures and Tables

**Figure 1:** Comparison between control and observation groups.

**Figure 2:** Comparison between the control group and observation group based on TNM staging of the tumor, tumor number, and American Society of Anesthesiologists.

**Figure 3:** Comparison between the control group and the observation group based on risks such as low risk, medium risk, and high risk.

**Table 1:** General information.

Groups		Control group	Observation group	*χ*2/*t*	*P* value
Cases		50	50		
Gender	Male	28	26	0.154	>0.05
	Female	22	24		
Age (average)		56.15 ± 6.15	56.78 ± 6.17	0.269	>0.05
TNM staging of the tumor (cases)	T1	16	18	0.628	>0.05
	T2	34	32		
Tumor number (cases)	Single	18	17	0.146	>0.05
	Multiple	32	33		
American Society of Anesthesiologists	Level I	26	23	0.418	>0.05
	Level II	24	27		
Tumor diameter (cm) (average)		2.07 ± 0.49	2.09 ± 0.43	0.172	>0.05

**Table 2:** Results of clinical indicators.

Groups		Control group	Observation group	*P* value
Operative blood loss (ml)		76.43 ± 10.53	55.72 ± 9.25	<0.05
Catheter indention time (h)		46.25 ± 5.07	28.30 ± 3.41	<0.05
Length of hospital stay (d)		6.58 ± 0.92	3.41 ± 0.85	<0.05
Obturator nerve reflex rate (n (%))		3 (6.00)	0 (0.00)	<0.05
Depth of pathological specimen	Deep muscular layer was reached	38 (70.00)	50 (100.00)	<0.05
	Deep muscular layer was not reached	15 (30.00)	0 (0.00)	
Postoperative recurrence rate (n (%))		12 (24.00)	1 (2.00)	<0.05

**Table 3:** Results of risk grade.

Groups	Low risk	Medium risk	High risk
Control group	19 (38.00)	21 (42.00)	10 (20.00)
Observation group	28 (56.00)	17 (34.00)	5 (10.00)
*χ* ^2^	0.195	0.048	0.134
*P* value	<0.05	<0.05	<0.05

**Table 4:** Results of immune function indicators.

Groups		Control group	Observation group	*P* value
CD4^+^	Before operation	42.25 ± 4.31	42.10 ± 4.26	>0.05
	2 h after operation	38.44 ± 3.20	35.02 ± 3.11	<0.05

CD8^+^	Before operation	25.03 ± 3.18	24.12 ± 3.25	>0.05
	2 h after operation	33.51 ± 4.04	28.35 ± 3.68	<0.05

CD4^+^/CD8^+^	Before operation	1.69 ± 0.15	1.72 ± 0.23	>0.05
	2 h after operation	1.03 ± 0.21	1.34 ± 0.18	<0.05

**Table 5:** Results of complication indicators.

Groups	Bladder perforation	Obturator nerve reflex	Bladder irritation
Control group	6 (12.00)	4 (8.00)	5 (10.00)
Observation group	1 (2.00)	1 (2.00)	2 (4.00)
*P* value	<0.05	<0.05	<0.05

## Data Availability

The data used to support the findings of this study are included within the article.

## References

[1] Zheng H. Li, R., Du L., Zhang S., Zhu C., Wei W., He J. (2021). Epidemic status and trend analysis of bladder cancer in China. *Chinese Journal of Oncology*.

[2] Mark J. R., Gelpi-Hammerschmidt F., Trabulsi E. J., Gomella L. G. (2012). Blue light cystoscopy for detection and treatment of non-muscle invasive bladder cancer. *The Canadian Journal of Urology*.

[3] Chou R., Selph S., Buckley D. (2017). Intravesical therapy for the treatment of nonmuscle invasive bladder cancer: a systematic review and meta-analysis. *The Journal of Urology*.

[4] Ehdaie B., Sylvester R., Herr H. W. (2014). Reply to donald L. Lamm and nilay M. Gandhi’s letter to the editor re: behfar ehdaie, richard sylvester, harry W. Herr. Maintenance Bacillus calmette-guérin treatment of non-muscle-invasive bladder cancer: a critical evaluation of the evidence. Eur urol 2013;64:579-85. *European Urology*.

[5] Saginala K., Barsouk A., Aluru J. S., Rawla P., Padala S. A., Barsouk A. (2020). Epidemiology of bladder cancer. *Medical Science*.

[6] Danforth K. N., Lee J. S., Luong T. Q. (2015). Treatment of non-muscle invasive bladder cancer. *Journal of Clinical Oncology*.

[7] Are B. M. (2012). New technologies for detection and treatment of non–muscle-invasive bladder cancer (NMIBC) so important? A plea for adoption by teaching programs to improve results after standard white light transurethral resection of NMIBC. *European Urology*.

[8] Annels N. E., Simpson G., Arif M. (2015). Oncolytic immunotherapy for the treatment of non-muscle invasive bladder cancer using intravesical coxsackievirus A21. *Journal for ImmunoTherapy of Cancer*.

[9] Sasaki B. R. D. S., Camargo G. C. D. A., Reis I. B., Dias Q. C., Duran N., Fávaro W. J. (2021). A potential new therapeutic option for the treatment of nonmuscle invasive bladder cancer: combination of intravesical oncotherad immunotherapy and platelet rich plasma (PRP). *Journal of Clinical Oncology*.

[10] Ossick M. V., Assalin H. B., Kiehl I. G. A. (2020). Carcinogenesis and Bacillus calmette-guérin (BCG) intravesical treatment of non-muscle-invasive bladder cancer under tryptophan and thymine supplementation. *Nutrition and Cancer*.

[11] GengAimin L. X. (2020). Effect of transurethral plasma acicular electrode enucleation in the treatment of non-invasive bladder cancer[J]. *Hainan Medical*.

[12] Chao L., Liao K., Dong W. (2019). Efficacy of transurethral holmium laser resection of bladder tumor versus electrotomy for non-muscular invasive bladder cancer. *Journal of Applied Cancer*.

[13] GuJunchao N. (2016). Progress in the diagnosis and treatment of urological diseases. *International Journal of Surgery*.

[14] Babayev A. B., Loran O. B., Kostin A. A., Seregin A. V., Dadashev E. O., Loshchenov V. B., Babayev A. B. (2020). Results of using domestic fluorescent video system in the diagnosis and treatment of non-muscle-invasive bladder cancer. *Onkologiya. Zhurnal imeni P.A.Gertsena*.

[15] Schooneveldt G., Geijsen E. D., Van Ommen F. (2015). PO-0727: thermophysical fluid modelling for loco-regional hyperthermia treatment of Non-Muscle Invasive Bladder Cancer. *Radiotherapy & Oncology*.

[16] Xiao M., Tang G., Liu J. (2018). Meta-analysis of the efficacy of tranurethral unipolar resection versus bipolar resection in the treatment of non-muscular invasive bladder cancer. *Journal of Fujian Medical University*.

[17] Steinberg R. L., Thomas L. J., O’Donnell M. A., Nepple K. G. (2015). Sequential intravesical gemcitabine and docetaxel for the salvage treatment of non-muscle invasive bladder cancer. *Bladder Cancer*.

[18] Shenping Z., Yang J. (2020). Effect of transurethral holmium laser resection on postoperative recovery and recurrence rate in patients with non-muscular invasive bladder cancer. *Shanxi Medical Journal*.

[19] Bryan R. T. (2012). Optimising existing therapeutic strategies for the treatment of non-muscle-invasive bladder cancer: the role of intensive neoadjuvant intravesical mitomycin C. *European Urology*.

[20] Masanski I. (2015). 42 Immediate results of surgical treatment of non-muscle-invasive bladder cancer using the new en bloc TUR BT. *European Urology Supplements*.

